# Circular RNA circFBXO11 modulates hepatocellular carcinoma progress and oxaliplatin resistance through miR‐605/FOXO3/ABCB1 axis

**DOI:** 10.1111/jcmm.15162

**Published:** 2020-03-28

**Authors:** Jin Li, Xiaoping Qin, Ruishan Wu, Li Wan, Liang Zhang, Rui Liu

**Affiliations:** ^1^ Department of Pain Management The First Affiliated Hospital of Jinan University Guangzhou China; ^2^ Department of Urology The First Affiliated Hospital of Jinan University Guangzhou China; ^3^ Department of Laboratory Guangdong Provincial Family Planning Science and Technology Research Institute Guangzhou China; ^4^ Department of Radiation Oncology Suining Central Hospital Affiliated Hospital of Chongqing Medical University Suining China

**Keywords:** ABCB1, circular RNA, FOXO3, hepatocellular carcinoma, oxaliplatin resistance

## Abstract

Increasing findings suggest the critical role of circular RNA (circRNA) in human cancer, and chemotherapy resistance is a poor prognostic factor for hepatocellular carcinoma (HCC). The function of circRNA in the HCC oxaliplatin (OXA) resistance remains largely unknown. In this study, we found that circRNA circFBXO11 was significantly up‐regulated in HCC tissues, and the circFBXO11 overexpression was associated with poor prognosis. CircFBXO11 was found to promote the HCC proliferation, cycle progress and OXA resistance. Mechanistically, circFBXO11 was predominantly localized in the cytoplasm and harboured the miR‐605, thereby targeting FOXO3 protein. Furthermore, FOXO3 targeted the promoter region of ABCB1 to accelerate its expression. In conclusion, this research reveals the role of circFBXO11/miR‐605/FOXO3/ABCB1 axis in the HCC OXA resistance, providing new insight for circRNA‐based diagnostic and therapeutic strategies.

## 1 INTRODUCTION

Hepatocellular carcinoma (HCC) is the most common type of malignant primary tumour with high lethality rate and recurrence.^1^, ^2^, ^3^ Current treatment status revealed that the prognosis of patients with HCC is an enormous challenge.^4^ Up to now, the complete surgical resection is the major potentially curative choice for HCC; however, the lack of reliably sensitive predictive markers makes the definite diagnosis at advanced stages.^5^, ^6^, ^7^ Although significant advances have been gained in surgery, chemotherapy and radiation therapy, the survival rate is not accompanied by distinct improvements.

Circular RNAs (circRNAs) are a novel class of non‐coding RNA (ncRNA) transcripts derived from back‐splicing. CircRNAs are characterized by the covalently closed continuous loop structure without a 5’‐cap and 3’‐poly A‐tail. The large proportion of circRNAs is originated from the exons of protein‐coding genes, while a few are generated by introns or exon‐introns. CircRNAs are much more stable as comparing to the linear RNAs transcripts and resistant to RNA enzyme decay, which makes circRNAs suitable for predictive marker.^8^, ^9^ For example, circRNA circSLC3A2 exhibits the oncogenic role in the HCC by sponging miR‐490‐3p/PPM1F axis.^10^ Circ‐10720 was positively promoted by the transcription factor Twist1 in HCC, which absorbs miRNAs that target vimentin, providing new insight for circular RNA‐based diagnostic and therapeutic strategies.^11^

Chemotherapy resistance is a significant factor for the recurrence and metastasis of HCC.^12^, ^13^, ^14^ Oxaliplatin (OXA)‐based systemic chemotherapy is increasing as the most critical clinical medicine for HCC at advanced stage, getting a vital breakthrough for the tumour chemotherapy.^15^, ^16^, ^17^, ^18^, ^19^ For example, OXA inhibits the proliferation and migration of HCC and GAS7C overexpression induces the apoptosis of HepG2 and MHCC‐97 H cells. GAS7C inhibition could reverse the anti‐cancer effect of OXA and represses the N‐WASP/FAK/F‐actin pathway.^20^

In the present research, we found a novel identified circRNA circFBXO11 (hsa_circ_0001001) in HCC tissue and cells. CircFBXO11 was generated from the exon 8‐11 of FBXO11 gene and significantly up‐regulated in HCC tissues, and the circFBXO11 overexpression was associated with poor prognosis. This research reveals the role of circFBXO11/miR‐605/FOXO3/ABCB1 axis in the HCC OXA resistance, providing new insight for circRNA‐based diagnostic and therapeutic strategies.

## 2 MATERIALS AND METHODS

### 2.1 Patient tissue samples

Human tumour and adjacent normal tissue specimens (Forty samples) were collected from patients with HCC who underwent surgical resection at First Affiliated Hospital, Jinan University, between May 2017 and January 2018. Tissue samples were snap‐frozen in liquid nitrogen after the resection for further analysis. The clinical research had been approved by the Human Ethics Committee of First Affiliated Hospital, Jinan University. Patients had signed the consent forms before surgery. The clinicopathological resource was shown in Table 1.

**Table 1:** Relationship of circFBXO11 level with HCC patients’ clinicopathological

Parameters		circFBXO11		*P*‐value
		Low (20)	High (20)	
Gender				
Male	24	11	13	.613
Female	16	9	7	
Age				
<50 y	22	11	11	.879
≥50 y	18	9	9	
Histological grade				
Well	13	6	7	.754
Moderately	17	9	8	
Poorly	10	5	5	
Tumour size				
<5 cm	13	5	8	.026*
≥5 cm	27	15	12	
Lymphatic metastasis				
Yes	24	11	13	.137
No	16	9	7	
TNM stage				
I‐II	15	6	9	.115
III‐IV	25	14	11	
AFP (ng/mL)				
<400	12	4	8	.032*
≥400	28	16	12	

Note

AFP, alpha‐fetoprotein; TNM, tumour‐node‐metastasis.

* *P* < .05.

### 2.2 Cell culture

Human HCC cell lines (HepG2, Hep3B, SMMC‐7721, Huh7) and normal liver cell lines (Lo‐2) were commercially provided by the Cell Center of Peking Union Medical College (Beijing, China). Cells were maintained in modified Eagle's medium (DMEM, Gibco) added with 10% foetal bovine serum (FBS) (FBS, Gibco), 100 U/mL penicillin and 100 mg/mL streptomycin. For the establishment of OXA‐resistant HCC cell lines, HepG2 cells were continuously exposed OXA with increasing doses. The OXA concentration was ranged low to high until that HepG2/OXA cells could grow stably in the medium with the indicated OXA concentration.

### 2.3 Transfection

The target sequences were synthesized by GenePharma, including sh‐circFBXO11, circFBXO11 overexpression plasmid, miR‐605 mimics and corresponding controls. CircFBXO11‐silenced HepG2/OXA cell and circFBXO11 overexpression HepG2 cells were constructed using shRNA lentiviral vector or overexpression plasmid. Lentiviral vector was commissioned by GeneChem (Shanghai Genechem). The miRNA mimics transfection was performed with Lipofectamine 2000 (Invitrogen) according to the manufacturer's protocol. The sequences were listed in Table S1.

### 2.4 RNA isolation and reverse transcription PCR

Total RNAs were extracted from HCC tissue or cells using TRIzol reagent (Invitrogen) according to the manufacturer's instructions. For reverse transcription, the TAKARA PrimeScript Kit (Takara) was used. For PCR, Real‐Time PCR System (Life Technologies) was used to measure the relative gene expression. GAPDH or U6 was set as an internal control for RNA or miRNA. The relative transcription level of target genes was detected by the 2^−ΔΔct^ method. The sequences were listed in Table S1.

### 2.5 Oxaliplatin sensitivity assay

About 1 × 10^4^ cells per well were seeded to the 96‐well plate. After 24‐h incubation, the cells were treated with grading doses (0, 0.5, 1, 2, 4, 8, 16, 32 μg/mL) of OXA. CCK‐8 agent (10 μL, Beyotime Institute of Biotechnology) was added to each well, and the optical density (OD) value was measured at 450 nm. Cells without drugs were set as control (100% survival) and were used to calculate the concentration of each chemotherapeutic drug (IC50).

### 2.6 Western blot analysis

The total protein of tissues or cells was extracted with the radioimmunoprecipitation assay (RIPA) lysis buffer (Solarbio Science Technology) in accordance with the instructions. Protein concentration was determined using the bicinchoninic acid (BCA) kit. The proteins were transferred to the polyvinylidene fluoride (PVDF) membrane and then blocked with non‐fat milk for 1 hour at room temperature. The member was incubated with the primary antibodies (anti‐FOXO3, Abcam, ab47285, anti‐ABCB1, Abcam, ab170904, 1:1000). The ImageJ software was used for protein quantification analysis according to the ratio of the grey value of control GAPDH band.

### 2.7 Flow cytometry analysis

After transfection of 48 hours, the Annexin V‐fluorescein isothiocyanate (FITC) and propidium iodide (PI) double staining kit (Becton Dickinson) were administrated for the apoptosis detection. After the centrifugation at room temperature, cells were resuspended with PBS and incubated with 5 mL Annexin V‐FITC under dark conditions. Early apoptotic cells and advanced apoptotic cells were calculated for the relative ratio of apoptotic cells. For the cycle analysis, cells were washed with phosphate‐buffered saline twice and stained with propidium iodide for 30 minutes. Cell cycle was analysed using a flow cytometer (FACScan, BD Biosciences) equipped with CellQuest software (BD Biosciences).

### 2.8 Subcellular fractionation location

The nuclear/cytosolic fractions were separated from HCC cells and then purified by the PARIS kit (Life Technologies) according to the manufacturer's manual.

### 2.9 Dual‐luciferase reporter assays

Dual‐luciferase reporter assay was performed to confirm the interaction within circFBXO11, miR‐605, FOXO3 and ABCB1. 3’‐untranslated region (3’‐UTR) of putative binding sites were cloned into the pGL3 plasmid (Ambion) named wild‐type (WT) and mutant (Mut). 293T cells were cotransfected with either pGL3‐FOXO3‐WT or pGL3‐FOXO3‐MUT reporter plasmids (120 ng) with miR‐605 mimic (40 nmol/L) or negative control using Lipofectamine 3000 (Invitrogen). The assays were performed with the dual‐luciferase assay kit (Promega) according to the manufacturer's instructions. The luciferase reporter assay was conducted using the dual‐luciferase reporter assay system (Promega), in accordance with the manufacturer's instructions.

### 2.10 Chromatin immunoprecipitation (ChIP)

ChIP assay was performed according to the EZ ChIP Chromatin Immunoprecipitation Kit (Millipore). In brief, the cross‐linked chromatin was sonicated into fragment (200 to 1000 bp). Anti‐FOXO3 antibody was used to precipitate the DNA fragments to construct the DNA‐protein complexes. Normal immunoglobulin G (IgG) was used as a negative control. The ChIP‐precipitated DNA was quantified by qRT‐PCR (Applied Biosystems).

### 2.11 In vivo mice xenograft

Nude mice (four‐week‐old, BALB/c nude mice) were purchased from Animal Slac Laboratory Animal Center and maintained under specific pathogen‐free condition. Suspended 5 × 10^6^ cells in 100 μL serum‐free DMEM were subcutaneously injected into the flanks of the mice. Tumour length and width were monitored once every three days following the formula: volume = length×width^2^ × 0.5. Tumour weight was measured after kill. All animal studies were approved by the Institutional Animal Care and Use Committee of First Affiliated Hospital, Jinan University.

### 2.12 Statistical analysis

All experiments data were generated from at least in triplicate using Windows SPSS 18.0 (SPSS Inc). The data are expressed as the mean ± SD. The between‐group variance was analysed with Student's *t* test or one‐way ANOVA. 0.05 was considered as statistical significance.

## 3 RESULTS

### 3.1 The high expression of circFBXO11 in HCC tissue and cells

To discover the potential differently expressed circRNAs in the HCC tissue, we performed the circRNA microarray analysis. CircRNA microarray unveiled that there were hundreds of circRNA with dysregulated expression in the HCC tissue as comparing to the normal control tissue (Figure 1A). Volcano plot illustrated the up‐regulated and down‐regulated circRNAs in the high‐throughput sequencing (Figure 1B). Schematic diagram revealed the genetic loci of circFBXO11 in the FBXO11 gene (Figure 1C). CircFBXO11 was generated from the exon 11 to the exon 8 by back‐splicing. Sanger sequencing confirmed the junction sites of exon 11 with exon 8 (Figure 1D). RT‐PCR showed that the circular transcript (circFBXO11) was much more stable than the linear transcript (FBXO11 mRNA), suggesting the resistivity ability of circFBXO11 (Figure 1E). In the HCC tissue, circFBXO11 was found to be highly expressed as comparing to the normal tissue (Figure 1F, Table 1). Prognosis analysis showed that these HCC patients with high circFBXO11 had lower survival rate (Figure 1G). In conclusion, these findings support that circFBXO11 is highly expressed in HCC tissue and cells.

**Figure 1:** circFBXO11 is highly expressed in HCC tissue and cells. A, CircRNA microarray unveiled the hundreds of circRNA with dysregulated expression in the HCC tissue as comparing to the normal control tissue. B, Volcano plot illustrated the up‐regulated and down‐regulated circRNAs in the high‐throughput sequencing. C, Schematic diagram revealed the genetic loci of circFBXO11 in the FBXO11 gene. D, Sanger sequencing confirmed the junction sites of exon 11 with exon 8. E, RT‐PCR showed the stability of circular transcript (circFBXO11) with the linear transcript (FBXO11 mRNA). F, RT‐PCR showed the circFBXO11 expression in the HCC tissue. G, Prognosis analysis showed the survival rate of HCC patients with high or low circFBXO11. Data are the means ± SD. **P < .01

### 3.2 circFBXO11 promotes the tumour progress and OXA resistance of HCC cells

In HCC cells, circFBXO11 expression was found to be highly expressed (Figure 2A). For the cellular experiments, circFBXO11 knockdown and overexpression transfection were constructed to silence and enhance its expression. RT‐PCR showed that circFBXO11 expression was highly expressed in the OXA‐resistant cells (HepG2/OXA) as comparing to normal cells (HepG2) (Figure 2B). The transfection of short hairpin RNA (shRNA) targeting the circFBXO11 could silence its expression (Figure 2C), and the transfection of overexpression plasmid enhanced circFBXO11 expression (Figure 2D). OXA sensitivity analysis by CCK‐8 assay showed that circFBXO11 knockdown down‐regulated the 50% inhibitive concentration (IC50) of HepG2/OXA cells, while circFBXO11 overexpression up‐regulated the IC50 of HepG2 cells (Figure 2E). Flow cytometry analysis revealed that circFBXO11 knockdown induced the G1/G0 phase arrest and the higher apoptotic rate, while circFBXO11 overexpression alleviated the cycle arrest and apoptosis (Figure 2F,G). In vivo heterograft mice assay indicated that circFBXO11 knockdown repressed the tumour growth (Figure 2H). Overall, data indicate that circFBXO11 promotes the tumour progress and OXA resistance of HCC cells.

**Figure 2:** circFBXO11 promotes the tumour progress and OXA resistance of HCC cells. A, RT‐PCR showed that circFBXO11 expression in HCC cells B, RT‐PCR showed the circFBXO11 expression in the OXA‐resistant cells (HepG2/OXA) and normal cells (HepG2). C, The transfection of short hairpin RNA (shRNA) targeting the circFBXO11 could silence its expression in HepG2/OXA cells. D, The transfection of overexpression plasmid for circFBXO11 in HepG2 cells. E, OXA sensitivity analysis by CCK‐8 assay showed the 50% inhibitive concentration (IC50) of HepG2/OXA cells and HepG2 cells. F, Flow cytometry analysis revealed the cycle arrest of HepG2/OXA cells and HepG2 cells. G, Flow cytometry analysis revealed apoptosis of HepG2/OXA cells and HepG2 cells. H, In vivo heterograft mice assay indicated the tumour growth of HepG2/OXA cells with circFBXO11 knockdown. Data are the means ± SD. **P < .01

### 3.3 miR‐605 acts as the target of circFBXO11

The subcellular distribution of circFBXO11 was detected using the subcellular fractionation location analysis, showing that circFBXO11 was distributed in the cytoplasmic portion (Figure 3A). To investigate the potential target for circFBXO11, the candidate miRNAs were tested using the RT‐PCR, indicating that miR‐605 was significantly dysregulated with the transfection circFBXO11 knockdown (Figure 3B). Bioinformatics tools (CircInteractome, https://circinteractome.nia.nih.gov/) indicated that miR‐605 shared the complementary binding sites with circFBXO11 (Figure 3C). Luciferase reporter assay showed that miR‐605 closely targeted with the circFBXO11 (Figure 3D). RT‐PCR illustrated that miR‐605 expression was higher in the OXA‐resistant cells (HepG2/OXA) as comparing to normal cells (HepG2) (Figure 3E). Clinically, the higher miR‐605 indicated the better survival rate of patients with HCC (Figure 3F). The relationship within miR‐605 and circFBXO11 indicated that miR‐605 was negatively correlated with circFBXO11 (Figure 3G). In conclusion, these findings suggest that miR‐605 acts as the target of circFBXO11.

**Figure 3:** miR‐605 acts as the target of circFBXO11. A, Subcellular fractionation location analysis showed the cytoplasmic or nucleus portion of circFBXO11. B, RT‐PCR showed the expression of potential target for circFBXO11. C, Bioinformatics tools (CircInteractome, https://circinteractome.nia.nih.gov/) indicated the complementary binding sites of miR‐605 with circFBXO11. D, Luciferase reporter assay showed the targeting of miR‐605 with circFBXO11. E, RT‐PCR illustrated the miR‐605 expression in OXA‐resistant cells (HepG2/OXA) and normal cells (HepG2). F, Survival rate of HCC patients with lower or higher miR‐605. G, The correlation between miR‐605 and circFBXO11 was calculated by Spearman's rank correlation coefficients. Data are the means ± SD. **P < .01

### 3.4 circFBXO11/miR‐605 targets FOXO3

The potential target of circFBXO11/miR‐605 axis was predicted using the StarBase database (http://starbase.sysu.edu.cn/) (Figure 4A). Luciferase reporter assay indicated that miR‐605 combined with the FOXO3 3’‐UTR wild‐type, instead of the mutant (Figure 4B). Then, the miR‐605 mimics transfection could reduce the FOXO3 mRNA (Figure 4C). Moreover, RT‐PCR showed that circFBXO11 knockdown decreased the FOXO3 mRNA level, and the circFBXO11 overexpression could up‐regulated the FOXO3 mRNA (Figure 4D). The relationship within FOXO3 and circFBXO11 indicated that FOXO3 was positively correlated with circFBXO11 (Figure 4E). In conclusion, these findings suggest that FOXO3 acts as the target of circFBXO11/miR‐605 axis.

**Figure 4:** circFBXO11/miR‐605 targets FOXO3. A, The potential target of circFBXO11/miR‐605 axis was predicted using the StarBase database (http://starbase.sysu.edu.cn/). B, Luciferase reporter assay indicated the luciferase activity of the transfection of miR‐605 and FOXO3 3’‐UTR wild‐type or mutant. C, RT‐PCR revealed the FOXO3 mRNA with miR‐605 mimics transfection or control. D, RT‐PCR showed the FOXO3 mRNA level with circFBXO11 overexpression or circFBXO11 knockdown transfection. E, The correlation between miR‐605 and circFBXO11 was calculated by Spearman's rank correlation coefficients. Data are the means ± SD. **P < .01

### 3.5 Transcription factor FOXO3 promotes ABCB1 transcriptional level

To investigate the possible regulation of circFBXO11/miR‐605/FOXO3 axis in the HCC OXA resistance, we found that the overexpression of transcription factor FOXO3 could promote the level of ABCB1 protein in the HCC cells (Figure 5A). Bioinformatics analysis found that FOXO3 harboured the binding sites on the ABCB1 gene promoter (Figure 5B). Luciferase reporter vectors for the assay were constructed, including wild‐type and the site‐mutant controls (Figure 5C). Results indicated that the binding of FOXO3 with first site (GTAAACA) had the significant difference for the activity (Figure 5D). Chromatin immunoprecipitation (ChIP) followed by PCR analysis indicated that the enrichment was higher in the FOXO3 antibody (Figure 5E). Public database (GEPIA, http://gepia.cancer-pku.cn/) illustrated that FOXO3 was positively correlated with the ABCB1 expression (Figure 5F). In conclusion, these findings suggest that transcription factor FOXO3 promotes ABCB1 transcriptional level.

**Figure 5:** Transcription factor FOXO3 promotes ABCB1 transcriptional level. A, Western blot indicated the ABCB1 protein in the HCC cells after the overexpression of transcription factor FOXO3. B, Bioinformatics analysis indicated the binding sites of FOXO3 on the ABCB1 gene promoter. C, Luciferase reporter vectors for the assay were constructed, including wild‐type and the site‐mutant controls. D, Luciferase reporter assay indicated the activity of the cotransfection of FOXO3 with first site (GTAAACA) and second site (GTAAATT). E, Chromatin immunoprecipitation (ChIP) followed by PCR analysis indicated the enrichment in the FOXO3 antibody or control. F, Public database (GEPIA, http://gepia.cancer-pku.cn/) illustrated the positive correlation with FOXO3 and ABCB1 expression. Data are the means ± SD. **P < .01

## 4 DISCUSSION

The increasing evidence demonstrates the critical role of circular RNA (circRNA) in the human cancer. In recent years, the biological functions of circRNA are gradually realized by researchers. Existing literature indicated that circRNA could regulate the proliferation, metastasis and multidrug resistance.^21^ Here, we investigate the role of novel identified circFBXO11 in the HCC OXA resistance and tumour progress.

In the HCC tissue, we screened the dysregulated circRNA using the circRNA microarray and found hundreds of up‐regulated or down‐regulated circRNAs. One novel circRNA was significantly up‐regulated as comparing to normal controls, whose functions were still unclear. Therefore, we tried to identify its deepgoing role in the HCC tumorigenesis. Clinically, the overexpression of circFBXO11 was correlated with the poor prognosis of patients with HCC. In the cellular investigation, circFBXO11 promoted the proliferation and cycle progression of HCC cells. Besides, circFBXO11 could also accelerate the OXA resistance. These findings suggested that circFBXO11 might act as the oncogenic element for the HCC tumorigenesis.

Although these finding illustrated the oncogenic role of circFBXO11, the mechanism by which circFBXO11 promoted the HCC OXA resistance is still unclear. The subcellular analysis found that circFBXO11 was mainly located in the cytoplasm. MiR‐605 was found to be the target of circFBXO11, and the miRNA could also target its downstream target FOXO3 mRNA 3’‐UTR. FOXO3 is a member of fork head protein family, as well as a critical transcription factor. In this research, we found that transcription factor FOXO3 could accelerate the transcriptional level of ABCB1, thereby promoting its protein product level. In conclusion, the circFBXO11/miR‐605/FOXO3/ABCB1 axis could regulate the HCC progress and OXA resistance.

Multidrug resistance is a huge obstacle for the HCC treatment.^22^ The role of circRNA in the cancer‐related multidrug resistance is still unclear.^23^, ^24^ For example, circRNA Cdr1as overexpression inhibits the ovarian cancer cell proliferation and promoted the cisplatin‐induced cell apoptosis by regulating the miR‐1270/SCAI signalling pathway.^25^ CircKDM4C is down‐regulated in breast cancer tissues and associated with poor prognosis and metastasis. CircKDM4C significantly represses breast cancer proliferation, metastasis and doxorubicin resistance in vitro and in vivo.^26^ In non–small‐cell lung cancer, circ_0076305 is elevated in NSCLC, and more significantly up‐regulated in DDP‐resistant tissues and cells, which regulates STAT3 expression via sponging miR‐296‐5p.^27^

In present research, our findings revealed the critical roles of novel circRNA circFBXO11 in the HCC tumorigenesis and OXA resistance. CircFBXO11 could promote the proliferation, cycle progress and OXA resistance. For the mechanism investigation, we found that ABCB1 acted as the downstream target of circFBXO11/miR‐605/FOXO3 axis. ABCB1, which is also known as MDR1 or P‐GP, participated in the multidrug resistance of HCC.

In conclusion, the study revealed the critical function of novel circFBXO11 in the HCC OXA resistance. CircFBXO11/miR‐605/FOXO3/ABCB1 regulates the HCC tumorigenesis and OXA resistance, providing new insight for circRNA‐based diagnostic and therapeutic strategies.

## CONFLICT OF INTEREST

All authors declare no conflicts of interest.

## AUTHOR CONTRIBUTION

JL, XQ and LZ are responsible for cellular experiments. RW and LW are responsible for data analysis. RL is responsible for management.

## Supporting information

Table S1
